The article "An Investigation and Analysis of College English Majors' Autonomous Learning Ability in Ubiquitous Learning Environment" was published in 2022. Journal: J Environ Public Health.

# An Investigation and Analysis of College English Majors' Autonomous Learning Ability in Ubiquitous Learning Environment

**DOI:** 10.1155/2022/9103148

**Published:** 2022-07-06

**Authors:** Tao Chen

**Affiliations:** School of Foreign Languages, Wuhan University of Science and Technology, Wuhan 430081, Hubei, China

## Abstract

In order to solve the problem that there are many places with poor learning ability of college English majors, this study conducts research, evaluation, and research on many places with poor learning ability. The independent learning ability of college students in different majors is obviously different, and majors affect the independent learning ability by 24.2%. Developing students' ability to succeed is a hot topic in teaching and learning. This study examines the self-learning ability of English majors in multiple subject areas by means of questionnaires and interviews. The study found that most UK adults had good self-control, but they showed improvements in self-planning, literacy and communication skills, and collaboration skills. The overall self-control ability is at a medium level and needs to be improved. At the same time, it discusses the necessity of improving learning ability and self-discipline in different learning environments, as well as strategies for improving academic ability, providing important guidance for supporting the academic development of the college new student. Compared with elementary and high school, the breadth and depth of knowledge acquired in school have expanded beyond textbooks. Classroom sound is fast and informative, requiring students to spend a lot of time after class to digest and understand. If students do not perform well in college, the process of assimilation and acquisition can be disrupted. In the case of data being cracked, it is difficult to meet the needs of work due to insufficient learning ability or even to meet the needs, which is based on improving the relationship. For example, it is critical to develop and enhance the ability of college students to succeed in a variety of settings.

## 1. Introduction

The student years are the best time to develop independent skills. Schools should not only continue to optimize their teaching environment but also focus on using technology-based teaching environments, such as online teaching and guidance, to not only improve students' independent learning skills but also to reduce carbon and develop their environmental awareness. Students with excellent self-directed skills are often enthusiastic about life and have a goodwill toward society. They are more likely to be involved in environmental activities and to motivate others to take part in them. By learning English, they can be more involved in international environmental platforms and play a greater role.

The article "An Investigation and Analysis of College English Majors' Autonomous Learning Ability in Ubiquitous Learning Environment" was published in 2022. Journal: J Environ Public Health.

As soon as the concept of independent education was put forward, it became an important value of education in many countries. China has also made confidence in the education revolution a key goal. The theme of the national medium and long-term education reform and development plan for 2010–2020 is to vigorously promote independent education, participatory education, and scientific education, lay a legal foundation for permanent public education, and build an educational community. The 2010–2020 National Medium and Long-Term Education Reform and Development Plan outlines that education is the key to education. Human resources are the main source of capital for China's economic and human development, and education is an important way to improve human resources. We must take students as an important role, and teachers must guide, provide students with activities to give full play to, support student development as the starting point and goal of all school activities, let all students improve actively and vividly, respect the right to education and the rights of students' physical development and mental health, and provide all students with an appropriate education. There are hundreds of millions of skilled workers, tens of millions of professionals, and many senior technicians. At present, there are two problems in the research on autonomous learning of college English: almost all the research studies applied to autonomous learning of college English are based on the principle of borrowing concepts from different subjects. Ethnic self-directed education and research do not define mission conditions. In college English teaching, most research focuses on how to improve the success of English students through the concept of instructional modification and instructional strategies. To date, there has been no academic work on improving English students' learning abilities by taking into account the development of college English literature. This study aims to make an effort and try both, as shown in Figure 1.

## 2. Literature Review

A large number of research experiments show that both humanistic pedagogy and constructivist pedagogy show that cultivating the potential of autonomous learning is a historical goal that modern education must achieve. The rapid development of society requires learners to adapt to the changing world of the future. The potential for independent learning is crucial. It can help students expand their life options, which are theoretically an important part of self-study. The rapid development of science and technology provides equipment for autonomous learning. The design and production of tape recorders, video recorders, and television sets make it possible for foreign language learners to learn the target material. Most of the free language learning centers created in Europe and America rely only on these materials. These programs and self-help centers have been extensively developed to provide language learning options. Students can take classes or special education classes depending on their circumstances. In particular, the rapid development of global computer networks has made distance learning and learning a reality. It also plays an important role in creating a language learning environment and promotes the development of autonomous language learning [1].

The article "An Investigation and Analysis of College English Majors' Autonomous Learning Ability in Ubiquitous Learning Environment" was published in 2022. Journal: J Environ Public Health.

From 1960 to 1970, Lin and Huang analyzed and researched the English autonomous learning ability of college freshmen. The analysis of disinformation mainly focuses on the definition, function, and role of disinformation and the relationship between disinformation and specific data, including the development and research of implicit curriculum [2]. Initially, based on theoretical concepts and arguments, he continued to develop his own interpretation, identify the relationship between false information and data, clarify, and develop his own theoretical system, with a focus on the United States, status from 1960 to 1970. Then, it developed rapidly in Europe, Asia, and Africa and created many scientific secrets. For example, Zhu and Fei established a theoretical school, which is a critical relational school, a clinical expression school, and a functional school [3]. During this period, Burns Sardone and Summary Jun conducted scientific research from different angles, including all kinds of confidential information, such as class secrets, documents hidden in teaching documents, hidden English passwords, and hidden experimental data [4]. From the first stage of research to the present, the research on implicit foreign learning materials has never stopped, and many scholars have emerged, such as Kalaee et al. [5].

On the basis of the present, this study puts forward the research on the self-learning capital of English for freshmen in different environments. The internal and external directions of foreign language learning are independently coordinated and determine the degree of recognition of foreign language learning [6]. The ability to use “external guidance” on a case-by-case basis to identify individualized education competencies will assist school policy, school management at all levels, administrators, academics, and educators working to improve students' knowledge and ability to learn independently. Carefully supervising the development of the external direction of autonomous learning and actively improving the environment and necessary equipment for autonomous learning can promote the design and development of learners' awareness of autonomous learning and autonomous learning ability [7].

The article "An Investigation and Analysis of College English Majors' Autonomous Learning Ability in Ubiquitous Learning Environment" was published in 2022. Journal: J Environ Public Health.

## 3. Research and Analysis on the Construction of College English Learning Environment

### 3.1. Research on Language Learning Strategies Based on Web-Based Autonomous Learning

In the 1980s, many foreign scholars studied academic science. Learners are trained in collaboration, which effectively helps learners to remember; at the same time, the combination of metacognition, knowledge, and effective training also attracts researchers [8]. However, with the rapid development of network technology, research on language learning strategies based on network autonomous learning has begun to attract foreign learners. The researchers say that learning a second language in the classroom requires the support of teachers themselves, and teachers should help students develop their experience by completing different tasks online [9].

### 3.2. Meaning of Autonomous Learning

Since the introduction of self-directed education, although there are more and more scholars, there has been no generally accepted comprehensive definition [10]. Professor Zimmerman, a famous American self-taught scholar, outlined three main points of self-study: motivation and attitude; self-education is a way of expressing self-esteem. It is believed that independent learners can monitor the benefits of their learning strategies and improve their learning based on this guidance; independent learners know when and how to use specialized learning strategies or respond appropriately [11]. Many domestic scholars believe that self-study generally has three main points: self-study is a synthesis of learners' abilities, learning attitudes, and educational strategies [12]. In fact, it can also be said that it is the learner's ability to guide and monitor their own learning and measure performance. Self-directed learning means that students freely choose their own educational goals, learning, learning, and learning content or are exempt from the free choice provided by the learning mechanism [13]. Self-directed education is a course in which specific learning goals are formulated according to the characteristics and needs of students or according to the teaching of teachers, and the learning goals are achieved through their personal efforts, as shown in Figure 2.

### 3.3. Autonomous Learning of College Students

The education of college students is different from primary and secondary schools and depends on teachers' planning and guidance. There are many student periods in universities, but more are acquired through student self-learning [14]. Self-directed learning provides options for college students. They can plan lessons according to their needs without affecting the lessons planned by teachers. When college students study problems by themselves, they need to acquire knowledge in various ways and find the answers to the problems. At this point, teachers should be very supportive of students' individual learning and provide students with additional training and support [15]. Therefore, what college students need for independent education is a kind of academic support. Self-directed learning can not only improve skills, improve students' college knowledge, and improve academic performance but also an important way for students to succeed, allowing college students to recognize their self-worth and promote their own development [16]. On the other hand, in the process of autonomous learning, college students take the initiative to set learning goals, use mobile devices to select appropriate resources, achieve goals, seek help from others through their own efforts or exchange learning, improve students' academic performance, improve their communication and coordination skills, and complete their major academic training. At the same time, also understand the school's personal training of students [17]. On the other hand, with the continuous improvement of society and the updating of knowledge, if students do not learn new skills to work after graduation, the experience educated in school is just far from being able to complete the work. Therefore, self-directed education is a course that college students should know about and a great way to improve themselves and their goals. Only by continuously learning new knowledge and skills, supporting and improving oneself, can we meet the needs of the society for art [18].

The article "An Investigation and Analysis of College English Majors' Autonomous Learning Ability in Ubiquitous Learning Environment" was published in 2022. Journal: J Environ Public Health.

### 3.4. Constraints of Autonomous Learning

The autonomous learning ability of college students refers to the ability to learn through their own attitudes, behaviors, and abilities. Behavior is an important factor in learners taking responsibility for their own learning, challenging, willing to change, and learning; behavior-specific, it includes supporting learning, sharing the benefits of learning, and self-fulfilling educational goals, with rules and regulations, and activities carried out. Demonstrate skills, the ability to practice skills, manage practice, and develop study plans. Self-directed learning and the ability to support further learning and interaction, so learning support is an important factor affecting learning ability [19]. From the perspective of learning theory and learning theory, Gu Shimin believes that the foreign languages that can be learned can be limited by direct and indirect effects. Other important aspects of curriculum development include materials and relationships, such as teacher level and skill level; internal orientation conditions include interests, ideas, and initiation 20. Therefore, it is necessary to focus on the development of external orientations of learning ability, improving environmental relationships and education resources to facilitate the formation and development of students' learning abilities. Other scholars believe that the factors affecting learning ability include research ability, collaboration ability, self-awareness, motivated learning, and metacognitive ability. In addition, educators play an important role in enhancing the academic ability of students. Evaluation of related studies [21] is given in Table 1.

## 4. Experiment and Research

### 4.1. Exploratory Factor Analysis of Questionnaire

Make key points of the measured data, subtract the values, and get the initial load matrix. Since there is a certain correlation between the lengths of the degrees of freedom, the rotation of the load matrix is obtained using the maximum difference. According to past experience and analysis, the number of events is determined according to the following criteria: type characteristic value > 1; each item contains at least 2 items; excluded content is easy to register. Finally, eight items were identified [22], as given in Table 2.

### 4.2. Quantitative Study on the Current Situation of College Students' English Autonomous Learning Ability

#### 4.2.1. Variance Contribution Rate of Each Dimension of the Current Situation of Students' English Autonomous Learning Ability

Square the loading value of each dimension for each dimension and then calculate the variance of each dimension. The difference of different sizes, according to the score, is education > self-discipline > learning motivation > student evaluation > communication ability, which shows that everything has different abilities and self-training performance. Learning strategies were the highest and coeducational abilities were the lowest [23], as given in Table 3.

#### 4.2.2. Lack of Learning Mobility

The results showed that 56.6% of the students believed that English was a good language and wanted to learn English well; 52.8% of the students believed that they could learn English well; 43.7% of the students said that they did not work in education due to unfortunate or difficult work, which shows that these students are not well-educated; 33.7% of students are worried about failing the exam, which shows that students still have a strong interest in English and confidence in learning English well. At the same time, many students are experiencing severe anxiety. However, we also see from the table that 60.0% of the students are unable to cooperate with the teacher in the classroom, which indicates their personal responsibility and the onset of negative emotions [24], as given in Table 4.

The article "An Investigation and Analysis of College English Majors' Autonomous Learning Ability in Ubiquitous Learning Environment" was published in 2022. Journal: J Environ Public Health.

#### 4.2.3. Basic Information of College Students

Key data for college students include gender, grade, and size. The special points are discussed as follows: among the respondents, 144 were girls, accounting for 46.15% of the total, and 168 were boys, accounting for 53.85% of the total. The distributions of the study data are equal, which suggests that random sampling is scientifically sound [25], as given in Table 5.

Among the respondents, there were 84 freshmen, accounting for 26.92% of the total; 105 graduates, accounting for 33.65%; 45 students, accounting for 14.42%; and 78 graduates, accounting for 25%. It can be seen that there are subtle differences between students, 12th graders, 12th graders, and adults, but there are fewer older students, affecting the majority of students. The data are completely similar, as given in Table 6.

#### 4.2.4. Analysis of the Relationship between Autonomous Learning and Traditional Teaching Elements

Although the curriculum has always been self-learning, even if the new classroom model is suitable for self-learning, the teacher's role in student learning, the average impact of self-learning is 3.07, slightly above average. 3 in total on average. It shows that most students believe that this teaching method has been unable to effectively improve students' interest in English autonomous learning. However, the benefits of new classroom models, such as group study and seminars, are less than ideal. The reason for the above phenomenon is that students often interpret self-study as their own autonomous learning while ignoring the importance of communication and participation. Participatory learning is an important way to learn autonomous English. Through the collaboration of students, we can not only exchange information but also supervise and compete with each other to improve the learning effect, as given in Table 7.

Guided by the required data, colleges and universities formulate college English teaching syllabus and college English teaching strategies according to the actual situation of the university, decompose the teaching objectives of the university, divide professional courses, and create professional courses. The syllabus usually specifies the teaching content, teaching and organization, and finally the selection of courses and the use of teaching as shown in Figure 3.

The article "An Investigation and Analysis of College English Majors' Autonomous Learning Ability in Ubiquitous Learning Environment" was published in 2022. Journal: J Environ Public Health.

Self-directed learning external supervision: self-directed learning supervision can be divided into self-directed learning and extracurricular activities according to the learning situation and objects of concern. Among them, external oversight includes academic support or accountability. The availability of external supervision is gradually reduced or even reversed to improve students' self-discipline and self-directed learning. As an important part of external supervision, supervising teachers play an important role in self-study. As a means of ensuring the effectiveness of classroom instruction, it prepares, evaluates, evaluates, delivers, and revises instructional activities throughout the process as shown in Figure 4.

### 4.3. Students Lack a Correct Understanding of Autonomous Learning Monitoring

Although most students know that college English education in the online environment must be influenced by all parties on campus, many students still think that self-directed education is self-employed and teachers should not interfere too much. 65% met the conditions, 52.8% generally met the conditions, and 12.2% of the students believed that teachers should not interfere too much. The above data show that students do not have a good understanding of autonomous learning in an online environment, which may have a certain impact on the assessment results, as given in Table 8.

### 4.4. Creation Principle of Innovative College English Grammar Teaching Derivation Formula

Through long-term college English grammar teaching, it is not difficult to find that there is a certain consistency in the principles of college English grammar itself. The concepts in each chapter of college English grammar are independent and interrelated, that is, the concepts before and after echo each other and do not exist independently. In particular, there are some common rules that are shared across multiple languages. After years of teaching research and practice, the author has finally found some moving texts of 16 timepieces, sounds, exemplars, and informal texts in college English grammar. They can be connected using designs. As long as people are familiar with these standards, they can identify the various concepts between them and thus develop this outline, which is called innovative college English grammar. The derivation formula is

(1) $$\begin{array}{c} \text{Aux}\cdot \left(1\right)+F\cdot V. \end{array}$$

For example, Wierzbicka believes that in order to show the exact meaning of “punishment,” we need to use the following event domain: *y* is punished because of *Z* as shown in the following equation.

(2) $$\begin{array}{c} X\left(\text{punish}\right)Y\left[\text{for}Z\right]\cdot =X. \end{array}$$

The article "An Investigation and Analysis of College English Majors' Autonomous Learning Ability in Ubiquitous Learning Environment" was published in 2022. Journal: J Environ Public Health.

### 4.5. Analysis of the Significance of Differences in the Passing Rate of CET4 in Countries

The 2013 and 2014 prices in a nonforeign language are two separate examples and the significance of the difference between these two rates is being tested. Key specification: if the key is set to 0.05, its theoretical Z value is 1.960. The test statistics assume that P1 = P2 or P1-P2 = 0, that is, there is no significant difference in the CET4 pass test between the two students. The passing score for nonforeign languages was P10 in 2004 and p in 2003. Here, we assume two equals the sum of all. At this time, regardless of whether there is an example of an equivalent model, the error calculation model is shown in the following equations.

(3) $$\begin{array}{c} \sigma_{Dp}=\sigma_{p1-p2}=\sqrt{\frac{\left(p1p2+n1n2\right)\left(n1q1+n2q1\right)}{n1n2\left(n1n2\right)}}, \end{array}$$

(4) $$\begin{array}{c} Z=\frac{\left(p1-p1\right)-0}{\sigma_{p1-p2}}=\frac{p1-p2}{\sigma_{p1-p2}}=2.72. \end{array}$$

Gunning entered advertising in 1935 and recently discovered that many high school graduates were unable to understand the content of a good newspaper. He explained the reason for this phenomenon because letters in newspapers are full of “clouds” (not necessarily hard). On this basis, it is decided to clarify the relationship between the text and the reader. He developed the nebulizer in his 1952 book The Technique of Clear Writing, which estimated the level of writing. For example, the barometer of text is 12, which means that American high school students can understand it, and the readability of Frog is expressed by the following equation.

(5) $$\begin{array}{c} 0.4=\left(X_{1}+X_{2}\right). \end{array}$$

The Flesch formula uses long words to determine how readable the reader is when understanding the words. Instead, Dale and Chall postulate that a word's readability depends on whether it is included in a list of words that 80% of fourth graders know and that words that are not in the correct word are considered “difficult words.” In 1948, they published Dale-Char's formula for readability in the article “Formulas for Predicting Readability,” where *X*_1_ is the average number of words in a sentence per 100 words, and *X* is the number of words greater than or equal to 3, as shown in the following equation.

(6) $$\begin{array}{c} 0.1579=X_{1}+0.0496X_{2}. \end{array}$$

Jing Xixing's research is based on the Chinese guide for primary and secondary schools in Taiwan, with a total of 12 grades. Each semester is used according to reading level, with a total of 24 levels. At the same time, it divides words into known words (such as Changyue) and unknown words. From readable options: all words, all sentences, and familiar words as

(7) $$\begin{array}{c} 1.1578=X_{1}+2.1497X_{2}. \end{array}$$

Sun Hanyin selected 20 Chinese articles with about 250 words each to conduct a Gestalt test for middle school students. Based on the extracted readability factors and test scores, he created the following formula:

(8) $$\begin{array}{c} 3.2578=X_{1}+3.2496X_{2}+2.486x_{3}^{1}. \end{array}$$

Erda of Fujian Normal University believes that the readability of English is determined by the readability of words and sentences. The legibility of English words is measured according to the order of words in the textbook. In this system, words are divided into eight levels. In the University Edition, the eight levels are the eight levels specified in the outline issued by the State Education Commission. Erda divides the length of English sentences into four categories. The length of these four types of sentences is 1–15 words in the first category, 16–25 words in the second category, 26–35 words in the third category, and 36 words or more in the fourth category. The readability ratio of vocabulary to sentence is calculated to be 9 : 1 by asking students to judge. The readability of text should know the values of at least 14 variables, as shown in the following formula.

(9) $$\begin{array}{c} \frac{0.9\left(1.25W1+2.5W2+3.75W3+5W4+6.25W5+7.5W6+8.75W7+10W8\right)}{W}+\frac{0.1\left(10S1+7.5S2+5S3+2.5S4\right)}{S}. \end{array}$$

In the study of the readability formula, Wang Lei further considers the types of words and Chinese sentence breaks and uses some other readability factors to construct a readability formula, including the number of words, simple words, function words, and clauses, as shown in the following formula.

(10) $$\begin{array}{c} \text{Readability}=72.748-0.462X_{1}+0.802X_{2}-7.515X_{3}+2.466X_{1}. \end{array}$$

Stenner, Smith, and Burdick (1983) analyzed more than 50 semantic variables and found that word frequency is the best operation for reading semantic components. Therefore, they chose two variables, word frequency and sentence length, to form their formula, as shown in the following formulas.

(11) $$\begin{array}{c} \text{The Lexile}=\left[\left(\text{Logit}+3.3\right)\times 180\right]+200, \end{array}$$

(12) $$\begin{array}{c} \text{Logit}=\left(9.82247X_{1}\right)-\left(2.14634X_{2}\right)-\text{constant}. \end{array}$$

The article "An Investigation and Analysis of College English Majors' Autonomous Learning Ability in Ubiquitous Learning Environment" was published in 2022. Journal: J Environ Public Health.

### 4.6. Adaptive Principle Analysis

In the adaptive model, writing the model, learning the model, and modifying the model are the three main modules. Therefore, Xahm describes the corresponding changes to the registration model, the design model, and the learning model, so that the rationale for using the change model in the model can be explained with more reason and clarity. About the preset mode, the compiler itself presets various themes according to different technologies, corresponding to the “preset” mode of EAC and PD. This “preset” isolation will create corresponding navigation lighting for users of various aluminum panels. Determine each lead plate group based on the average result of the shortest path, the average length of the shortest path, and the number of lines of the desired graph, as shown in the following equation.

(13) $$\begin{array}{c} S\left(k\right)=\frac{\beta_{0}\mu \left(k\right)+\beta_{1}n\left(k\right)+\beta_{2}p\left(k\right)}{\beta_{0}+\beta_{1}+\beta_{2}}. \end{array}$$

Learner model: the learner model can be updated every time the learner requests a link. Of course, the update frequency or time interval can also be customized. When the learner passes through a specific path ruler and requests the next node RR, the degree of coupling between the learner and each lead plate category is judged according to the probability that the ruler belongs to the domain path corresponding to a lead plate category *K*, the probability of selecting the next node R through this path, and the time spent in the domain path corresponding to each lead plate category *K*, as shown in the following formula.

(14) $$\begin{array}{c} d\left(k\right)=\frac{\alpha_{0}c\left(k\right)+\alpha_{1}r\left(k\right)+\alpha_{2}t\left(k\right)}{\alpha_{0}+\alpha_{1}+\alpha_{2}}. \end{array}$$

Overall model: according to the user's initial lead plate type, the user's current lead the plate membership model a (*k*), and (*k*), and D (*k*), determine which lead plate type the user should give, and recommend the domain learning path corresponding to this lead plate type to him/her, as shown in the following formula.

(15) $$\begin{array}{c} A\left(k\right)=\frac{\gamma_{0}A_{0}\left(k\right)+\gamma_{1}A\left(k\right)+\gamma_{2}d\left(k\right)+\wedge \gamma_{3}s\left(k\right)}{\gamma_{1}+\gamma_{2}+\wedge \gamma_{3}}. \end{array}$$

Xahm's learning standards are generally considered to be based on knowledge level, learners' educational data, and considerations of saving and checking time. On the basis of the curriculum, we add concepts such as skills, standards, environment, and curriculum, which will help create a better learning environment. Knowledge level refers to the advanced level of all knowledge in the registration system, which is the process of competitive pricing.

(16) $$\begin{array}{c} \text{knowledge Level}=\left\{\left(k_{1},h_{2}\right)Ik,\in AD,h,\in H\right\}. \end{array}$$

The article "An Investigation and Analysis of College English Majors' Autonomous Learning Ability in Ubiquitous Learning Environment" was published in 2022. Journal: J Environ Public Health.

### 4.7. Current Situation and Characteristics of College Students' Autonomous Learning Ability

In order to determine the critical state of college students' learning self-efficacy, a statistical analysis of the mean and standard deviations of college students' autonomous learning ability and its dimensions was carried out. The specific results are given in Table 9.

#### 4.7.1. Differences in Self-Directed Ability

To determine differences in behavioral potential among students of different genders, grades, and sizes, this study made model D experiments independent and one-way. ANOVA was performed on the behavioral potential of college students of opposite sex, grade, and size. Detailed study results are given in Tables 10–12.

#### 4.7.2. Differences in Self-Selection Ability

In order to determine the differences in the self-selection potential of college students by gender, grade, and size, this study made the model D experiment independent and one-way, and the analysis of variance of college students selected the self-potential of gender, grade, and size. Detailed study results are given in Tables 13–15.

This study will use the potential of self-study and its length as a distinction between college students and college students as an independent exchange of ANOVA methods. Different majors have different self-learning abilities, and majors have a 24.2% impact on proficiency. In various fields of learning ability, there are significant differences in the product distribution of behavioral ability, self-selection ability, self-control ability, and self-discipline ability. After many comparisons, it is found that in terms of behavioral ability, self-selection ability, and self-control ability, students' pressure on information and history is greater than that in science and engineering and art, but in terms of personal potential. Art college students are not just literature and historical art. Majors described 27.5% change in self-efficacy, 26.7% change in self-efficacy, 16.4% change in self-efficacy, and 12.4% change in self-efficacy.

(17) $$\begin{array}{c} \sigma_{DP}=\sigma_{p1-p2}=\sqrt{\frac{\left(n1p1=n2p2\right)\left(n1q2+n2q2\right)}{n1n2\left(n1+n2\right)}}=0.058. \end{array}$$

## 5. Conclusion

The four main definitions of self-directed education are that the purpose and form of self-directed education are different at different stages of development, the environment in which self-directed education occurs is also quite different, and the degree of self-government also has many differences. The data reflection of self-learning also reveals many characteristics. The interplay of these events makes it difficult for scientists to agree on the meaning of autonomous learning. Therefore, there is a conflict between the “status view” of foreign independent education, the “potential view” of foreign independent education, and the “psychological view” of independent study abroad. The “approval” of foreign independent education, the “environmental view” of foreign independent education, the “potential” learning of independent education, and the “critique” of independent learning of foreign education are harmonious. The characteristics of Chinese foreign language education are “see” and “see.” We discuss the impact of the external social environment and objective data on learning from the perspective of the relationship between learning and the environment. The ability to use “outreach” means more self-learning, and self-directed learning means the type of cognition and ability that learners engage in language learning and desire to take responsibility for their own language learning; the ability to apply effective language learning strategies and the ability to develop the material and relationships that foreign language learners need to become proficient in the language. This is the first new advance in this study and the basis for all studies. It is the responsibility of students to adapt freely to the external environment, overcome the negative effects of learning English as a foreign language in China, create the best second language learning environment, and improve the achievement and effectiveness of autonomous English learning. However, learners face the main role of being a human being when their abilities are insufficient. In language learning, schools, communities, governments, schools, and educators have a responsibility to play a key role in improving the quality of learning and creating an enabling environment. Learn languages, better integrate into students' internal environment, socialize, and promote growth. Ability to study independently abroad. How to improve external guidance by creating English language courses, create a good English language environment for English learners, improve the nature of knowledge and skills of self-study, and support the completion of college English courses are the key issues that this research strives to solve and address solution.

The article "An Investigation and Analysis of College English Majors' Autonomous Learning Ability in Ubiquitous Learning Environment" was published in 2022. Journal: J Environ Public Health.

## Figures and Tables

**Figure 1:** The independent learning ability of college English major freshmen.

**Figure 2:** Published annual trend chart.

**Figure 3:** English syllabus.

**Figure 4:** Activity plan.

**Table 1:** Statistics of factors restricting autonomous learning ability.

Serial number	Author	Year	Restrict autonomous learning ability
1	Candy	1990	Internal characteristics
2	Bincp	1990	Personal characteristics, self-setting goals
3	Gamson	1996	Emotion, self-monitoring ability
4	Riedp	2000	Autonomous learning ability is manifested in attitude
5	Chen Shihong	2001	Objective factor
6	Feng Lvquan	2001	Information ability

**Table 2:** Exploratory factor analysis.

Title number	Project	Common degree	Factorload
Factor	The contribution rate of learning strategies (eigenvalue is 1.08) is 12.265		
24	When learning English, try to combine what you usually learn with your existing knowledge	616	650
18	In order to improve their English communication level, I take advantage of various opportunities to train myself	682	542
25	Be able to grasp the key points in listening to English class	544	532
19	Understand the teaching objectives and requirements of teachers in each class	516	554

**Table 3:** The variance contribution rate of each dimension.

Learning strategy	Learning motivation	Self-management	Student information ability	Teacher information ability	Information resources	Student evaluation	Assist in communication ability
12.263	5.332	6.882	5.103	4.962	4.574	4.023	3.864

**Table 4:** Learning motivation.

Project	Topic content	Title number	Never	Sometimes	Often	Always
Interest	Feel interested in English	6	9.6	31.2	25.4	19.6
Self-efficacy	English test anxiety	9	7.8	33.2	29.5	5.3
	Believe I can learn English well	10	9.3	34.5	30.6	21.3
Subject consciousness	Actively participate	9	8.5	36.5	31.2	6.3

**Table 5:** Gender distribution of college students.

Category	Name	Number of people	Percentage (%)
Gender	Male	158	53.85
	Female	133	46.15

**Table 6:** Grade distribution of college students.

Category	Name	Number ofpeople	Percentage (%)
Grade	Freshman year	74	23.96
	Sophomore year	103	33.64
	Junior college	39	36.22
	The fourth year of college	69	25.33

**Table 7:** Descriptive statistics.

	*N*	Minimum	Maximumvalue	Meanvalue	Standard value
t24	215	0	4	3.04	1.222
t25	215	0	4	3.06	1.065
t26	215	0	4	2.26	1.325
t27	215	0	4	2.35	1.036
Valid *N*	215				

**Table 8:** Questionnaire on students' awareness of autonomous learning monitoring.

	Number of people	Percentage (%)
Not suitable at all	15	7.6
Usually not suitable	36	21.1
Sometimes suitable	14	6.3
Usually suitable	23	12.1
Perfect fit	94	52.1

**Table 9:** Distribution of college students' autonomous learning ability.

	Self-orientation	Self-selection ability	Self-regulation ability	Self summarizing ability	Autonomous learning ability
Mean value	3.1888	3.2455	3.3220	3.1240	3.1200
Standard deviation	0.7365	0.7750	0.7561	0.7356	0.6236

**Table 10:** Comparison of differences in self-orientation ability of college students of different genders.

Dependent variable	Gender	Number	Mean value	Standard deviation	*T* value	*N*2
Self-orientation	Male	167	3.0354	0.76452	−0.3014	0.039
	Female	134	3.3640	0.54688		

The article "An Investigation and Analysis of College English Majors' Autonomous Learning Ability in Ubiquitous Learning Environment" was published in 2022. Journal: J Environ Public Health.

**Table 11:** Comparison of self-orientation ability of college students in different grades.

Dependent variable	Grade	Number	Mean value	Standard deviation	*F*	Multiple comparison	Correlation strength
Self-orientation	Freshman	83	3.1330	0.6345			
	Sophomore	106	3.0366	0.5675	27.81	4 ＞ 1 ＞ 3	0.164
	Junior	44	3.1667	0.4354			
	Senior	76	3.3456	0.5637			

**Table 12:** Comparison of self-orientation ability of college students in different majors.

Dependent variable	Major	Number	Meanvalue	Standard deviation	*F*	Multiplecomparison	Correlationstrength
Self-orientation	Literature and history	125	3.142	0.7602	10.56	2 ＞ 3 ＞ 4	0.253
	Science and engineering	152	3.126	0.7423			
	Arts	24	3.392	0.7452			

**Table 13:** Comparison of self-selection ability of college students of different genders.

Dependent variable	Gender	Number	Mean value	Standard deviation	*T* value	*N*2
Self-selection ability	Male	165	3.212	0.845	−3.212	0.032
	Female	133	3.214	0.625		

**Table 14:** Comparison of self-selection ability of college students in different grades.

Dependent variable	Grade	Number	Mean value	Standard deviation	*F*	Multiple comparison	Correlation strength
Self-selection ability	Freshman	83	3.124	0.425			
	Sophomore	104	3.214	0.345	40.61	3 ＞ 4 ＞ 1	0.156
	Junior	43	3.124	0.654			
	Senior	76	3.456	0.745			

**Table 15:** Comparison of self-selection ability of college students of different majors.

Dependent variable	Major	Number	Meanvalue	Standard deviation	*F*	Multiple comparison	Correlation strength
Self-selection ability	Literature and history	165	3.212	0.786	32.64	4 ＞ 2 ＞ 3	0.113
	Science and engineering	154	3.542	0.674			
	Arts	22	3.458	0.825			

## Data Availability

The dataset used to support the findings of this study is available from the corresponding author upon request.
